# Clearance Rate and BP-ANN Model in Paraquat Poisoned Patients Treated with Hemoperfusion

**DOI:** 10.1155/2015/298253

**Published:** 2015-01-28

**Authors:** Lufeng Hu, Guangliang Hong, Jianshe Ma, Xianqin Wang, Guanyang Lin, Xiuhua Zhang, Zhongqiu Lu

**Affiliations:** ^1^Department of Pharmacy, The First Affiliated Hospital of Wenzhou Medical University, Wenzhou 325000, China; ^2^Department of Emergency, The First Affiliated Hospital of Wenzhou Medical University, Wenzhou 325000, China; ^3^Function Experiment Teaching Center, Wenzhou Medical University, Wenzhou 325035, China

## Abstract

In order to investigate the effect of hemoperfusion (HP) on the clearance rate of paraquat (PQ) and develop a clearance model, 41 PQ-poisoned patients who acquired acute PQ intoxication received HP treatment. PQ concentrations were determined by high performance liquid chromatography (HPLC). According to initial PQ concentration, study subjects were divided into two groups: Low-PQ group (0.05–1.0 *μ*g/mL) and High-PQ group (1.0–10 *μ*g/mL). After initial HP treatment, PQ concentrations decreased in both groups. However, in the High-PQ group, PQ levels remained in excess of 0.05 *μ*g/mL and increased when the second HP treatment was initiated. Based on the PQ concentrations before and after HP treatment, the mean clearance rate of PQ calculated was 73 ± 15%. We also established a backpropagation artificial neural network (BP-ANN) model, which set PQ concentrations before HP treatment as input data and after HP treatment as output data. When it is used to predict PQ concentration after HP treatment, high prediction accuracy (*R* = 0.9977) can be obtained in this model. In conclusion, HP is an effective way to clear PQ from the blood, and the PQ concentration after HP treatment can be predicted by BP-ANN model.

## 1. Introduction

Paraquat (1,1′-dimethyl-4,4-bipyridinium dichloride, PQ) is a widely used nonselective herbicide. It has been detected in many fruits such as olives, onions, tomatoes, corn, and also in many vegetables [1]. Although the use of paraquat is safe for routine agricultural purposes, PQ is highly toxic to many human and animal organs [2]. Extensive studies have demonstrated that people exposed to PQ have a higher risk of developing Parkinson's disease and neurotoxicity [3–5]. Most importantly, PQ has a high rate of mortality that is 60–70% [6]. Acute ingestion of PQ 20–40 mg/kg (7.5–15.0 mL of 20% (w/v) PQ concentrate) can cause serious symptoms such as liver, lung, heart, and kidney failure within several days and lead directly to death [7]. Without prompt treatment, the survival rate of PQ toxicity is about 13% [8].

The mechanism of PQ intoxication is associated with accumulation of reactive oxygen species (ROS) and toxic free radicals that cause multiorgan failure with circulatory collapse and pulmonary fibrosis with respiratory failure [9, 10]. Therefore, the current therapeutic procedures of PQ poisoning mainly include diminishing absorption of PQ in the gastrointestinal tract, increasing elimination of PQ from the body, administration of antioxidants, and the maintenance of vital functions [8, 11].

Hemoperfusion (HP) is commonly conducted using activated charcoal and resin, which is effective for clearing protein-bound, lipid-soluble drugs and small water-soluble molecules. HP is the most effective way to eliminate PQ from blood, which is an important factor related to prognosis [12]. A large-scale retrospective cohort study reveals that early HP treatment can reduce mortality [13] and significantly improve outcomes for PQ-poisoned patients [11].

However, being an extracorporeal form of treatment, HP can result in a series of complications. The most dangerous side effect is platelet depletion. Other side effects include charcoal embolism, leukopenia, fibrinogenopenia, and hypocalcemia [14]. In addition, HP treatment is expensive and patients can easily become infected with blood-transmitted diseases [15]. Therefore, it should be administered with the appropriate strategy and at the appropriate time.

In order to assess the validity of HP treatment for blood clearance of PQ and to ensure timely and proper treatment, this study investigated patients with acute PQ intoxication who received HP. The plasma PQ concentration was determined by a simple, rapid, and inexpensive HPLC method. The clearance rate of PQ was calculated by plasma PQ concentrations before and after first HP treatment. And a prediction model was developed by artificial neural network. The artificial neural network is a form of artificial intelligence which can mimic the human brain's data process [16]. It has been a very powerful modeling tool and widely applied to medical area such as predicting the plasma concentration of drugs, pharmaceutical properties of dosage forms, pharmacokinetics of antibiotics, and screening risk factors related to liver diseases [17]. In this study, we apply artificial neural network modeling to predict PQ concentration after HP treatment.

## 2. Materials and Methods

### 2.1. Chemicals and Reagents

PQ (purity > 98%) and 5-bromouracil (purity > 98%), as internal standard (IS), were purchased from Sigma-Aldrich Shanghai Trading Co. Ltd. HPLC grade methanol and acetonitrile were purchased from Merck Company (Darmstadt, Germany) and sodium dodecyl sulfate (SDS) was purchased from Shanghai Biological technology Co. Ltd. (Shanghai, China). Ultrapure water was prepared by a Millipore Milli-Q purification system (Bedford, MA, USA). All other chemicals were of analytical grade and used without further purification.

### 2.2. Instruments

For laboratory assessments, this study incorporated the use of a centrifuge (Beckman Coulter Inc., 21R), analytical balance (Mettler-Toledo International Inc.), Agilent 1260 Infinity HPLC system equipped with an on-line degasser, a quaternary pump, an autosampler, a thermostat-columned compartment, and a diode-array UV detector controlled by ChemStation.

### 2.3. Determination of PQ

#### 2.3.1. Analytical Conditions

An Agilent Zorbax HC-C_18_ (2.1 mm × 150 mm, 5 *μ*m) column was used for chromatographic separation with temperature set at 30°C. An isocratic elution programmed with mobile phase A (96%) and mobile phase B (acetonitrile, 4%) was conducted for chromatographic separation with a flow rate of 1 mL/min. Mobile phase A contained 20 mM sodium dihydrogen phosphate and 0.4 mM sodium heptanesulfonate. The pH was adjusted to 2.3 with phosphoric acid. The detection wavelength was 258 nm for both PQ and IS.

#### 2.3.2. Sample Preprocessing

Before sample extraction, 20 *μ*L of IS working solution (100 *μ*g/mL) was added to a 1.5 mL centrifuge tube which contained 200 *μ*L of plasma sample, followed by the addition of 100 *μ*L trichloroacetic acid–methanol (9 : 1, v/v). After the tubes were vortex mixed for 0.5 min, they were centrifuged at 14,900 g for 10 min. After mixing, the supernatant (10 *μ*L) was injected into the HPLC for analysis.

#### 2.3.3. Calibration Curves

Calibration curves were constructed. Eight calibration standards (0.05, 0.1, 0.25, 0.5, 1, 2.5, 5, and 10 *μ*g/mL) were prepared by spiking blank human plasma with appropriate amounts of the working solutions of PQ. Peak area ratios of PQ to IS were plotted against analyte concentrations. The standard curves were assessed by the equations for linear regression with a weighting factor of the reciprocal of the concentration (1/*x*) in the concentration range of 0.05–10 *μ*g/mL. The lower limit of quantification (LLOQ) was defined as the lowest concentration according to calibration curves.

#### 2.3.4. Precision and Accuracy

Precision and accuracy were assessed by the determination of quality control (QC) samples (0.08, 0.8, and 8 *μ*g/mL) in five replicates. Precision was subdivided into intraday and interday precision. The intraday precision measured the QC samples within a day while interday precision was measured within three days. The precision was expressed by relative standard deviation (RSD). The accuracy evaluated by the recovery was expressed by relative error (RE).

### 2.4. PQ-Poisoned Patients

This study was approved by the Medical Ethics Committee of the First Affiliated Hospital of Wenzhou Medical University and was conducted in accordance with the Declaration of Helsinki. The patients with a history of direct contact of PQ poisoning were involved in this study. All individual information of PQ-poisoned patients was securely protected and only available to the investigators. All data was analyzed anonymously.

### 2.5. Hemoperfusion Treatment

All PQ-poisoned patients, when PQ-poisoned (PQ > 0.05 *μ*g/mL) was confirmed, received active charcoal HP therapy in the emergency intensive care unit (EICU). HP was administered through femoral venous catheters at a blood flow rate of 200 mL/min. A single-use HA230 resin hemoperfusion apparatus (Zhuhai Jianfang Biotechnology Co., Ltd., Guangdong, China) was used which consisted of polypropylene housing material, cellulose, and activated charcoal adsorbent. After HP treatment, plasma PQ concentrations were dynamically monitored. Based on PQ concentrations, other conventional treatments were administered based on PQ-poisoned patient's symptoms.

### 2.6. Clearance Rate and Model

The clearance rate of PQ was calculated. Based on the clearance rate calculations, the clearance model of PQ was developed. The data of PQ concentrations from first HP treatment was loaded into the BP-ANN and established at MATLAB R2011a. PQ concentrations before and after first HP treatments were selected as the input layer and output data. The node numbers of hidden layer were based on the formula of $m=\sqrt{n+l}+a$, where *m* is the number of the nodes in the hidden layer, *n* is the number of nodes in the input layer, *l* is the number of nodes in the output layer, and *a* is a constant from 1 to 10 [18]. The transfer function of the hidden layer and output layer nodes was tansig and purelin; the training goal was set at 0.0015. The developed BP-ANN model of PQ was also used to predict the increased PQ concentration after first HP treatment. The PQ concentrations after first HP treatment were selected as the input layer and PQ concentrations before second HP treatments were selected as the output data.

## 3. Results

### 3.1. Determination of PQ

#### 3.1.1. Calibration Curve and Selectivity

There were good linear regressions of the peak area ratios versus concentrations in the concentration range 0.05–10 *μ*g/mL for PQ. Typical equation of the calibration curve was *y* = (0.3907 ± 0.0028)*x* + (0.0031 ± 0.0007), *r* = (0.9992 ± 0.0007), where *x* represented the ratios of PQ peak area to that of 5-bromouracil (IS), and *y* represented the plasma concentration. The LLOQ of PQ in plasma was 0.05 *μ*g/mL. The limit of detection (LOD) of PQ in plasma was 0.01 *μ*g/mL defined as a signal/noise ratio of 5. No interfering endogenous substance was observed at the retention time of the PQ and IS.

#### 3.1.2. Precision and Accuracy

The measured concentrations of PQ for each QC sample (0.08, 0.8, and 8 *μ*g/mL) for intraday and interday were listed in Table 1. The accuracy of three QC samples at each concentration, all less than 15%, was calculated by RSD. The precision of the method was calculated by RE at each QC sample. The assay performance data of precision and accuracy are presented in Table 1. The RSD of IS (0.5 *μ*g/mL) was less than 10% and RE ranged from −1.18 to 3.5. These results indicate that the method was satisfactory with respect to both accuracy and precision.

### 3.2. Characteristics of PQ-Poisoned Patients

There were 82 patients, hospitalized from March 1, 2012, to April 30, 2014, who had a history of direct contact with PQ. Among them, the PQ concentrations were under 0.05 *μ*g/mL in 38 patients. Three of them had extremely high, fatal plasma PQ concentrations, in excess of 50 *μ*g/mL and died quickly. A total of 41 patients met the inclusion criteria and were involved in this investigation. According to the PQ concentration in plasma before HP treatment, they were divided into two groups: Low-PQ group (0.05–1.0 *μ*g/mL, 9 males and 8 females) and High-PQ group (1.0–10 *μ*g/mL, 14 males and 10 females). The ages of PQ-poisoned patients ranged from 15 to 64.

### 3.3. HP Treatment of PQ-Poisoned Patients

All PQ-poisoned patients received HP treatment within 4 hours. In Low-PQ group, the PQ concentrations of most PQ-poisoned patients were below LLOQ after the first HP treatment. However, in High-PQ group, the PQ concentration was still over 0.05 *μ*g/mL. There is high correlation (*R* ^2^ = 0.8504) before and after first HP treatment in the two groups; the PQ concentrations profile is shown in Figure 1.

After first HP treatment, the PQ-poisoned patients in Low-PQ group had not received HP treatment again. In High-PQ group, 9 PQ-poisoned patients accepted second HP treatment within 24 hour, whose PQ concentrations were all slightly increased after first HP treatment (Figure 2). 5 PQ-poisoned patients, whose PQ concentrations still over 3.5 *μ*g/mL after first HP treatment, were aggravated quickly and given up the treatments. The other 10 patient received further treatment after 24 hour.

### 3.4. PQ Clearance Rate and BP-ANN Model

According to the PQ concentrations obtained from first HP treatment, the clearance rate of PQ in plasma was 73 ± 15%. And there was no statistical differences between male and female (*P* > 0.05). The clearance rate of PQ after second HP treatment was 73 ± 13%. There was no statistical difference for clearance rate of PQ between the first and second HP treatment (*P* > 0.05).

The BP-ANN clearance model of PQ quickly reached the training goal at epoch 157 (Figure 3). Mean square error (MSE) was 1.49 × 10^−3^, magnitude of the gradient was 1.93 × 10^−3^, number of validation checks was 0, and the correlation coefficient was 0.9977. The MSE is the average squared error between the network outputs and the target, which is the default performance function for feed-forward networks [19]. The correlation coefficient was used to assess the relationship between the outputs and the targets [20]. According to the developed BP-ANN model, the predicted PQ concentrations of 41 PQ-poisoned patients after first HP treatment were generated and were in agreement with measured PQ concentrations (Figure 4).

Based on the parameters of developed BP-ANN clearance model of PQ, the increased PQ concentrations after HP treatment were also predicted. These results showed there was also high correlation *R* = 0.9993, MSE was 3.96 × 10^−4^, magnitude of the gradient was 1,14 × 10^−2^, and the number of validation checks was 0.

## 4. Discussion

### 4.1. Determination of PQ in Human Plasma

The plasma PQ level is a key predictor of clinical outcome for PQ-poisoned patients. Determination of plasma PQ concentrations is necessary for treatment. PQ can be separated by HPLC using methanol [21], acetonitrile [22], or ion pairing agents [10]. We found that a combination of 0.2 M sodium hydrogen phosphate (pH 2.3) and acetonitrile, in a ratio of 96 : 4 (v/v), was the most suitable condition for separating PQ and IS. The retention time of PQ and IS was 5.9 min and 4.1 min, respectively, which was shorter than other reported HPLC methods [10, 21–23]. Several procedures, such as ion-pair liquid-liquid extraction and solid-phase extraction [21, 24], have been used for sample preparation. Herein, we used one step protein precipitation by combining trichloroacetic acid and methanol (9 : 1, v/v) that greatly shortened the time of analysis.

Various methods have been developed to analyze PQ in plasma such as capillary electrophoresis (CE) [25, 26], GC-mass-spectrometry (MS) [27–30], and HPLC-MS [31, 32]. HPLC is accurate, simple, rapid, inexpensive, and more suitable for dynamic monitoring of plasma PQ level [22].

### 4.2. HP Treatment in PQ-Poisoned Patients

As a rule, there are three methods used to remove PQ from the blood which include forced diuresis, hemodialysis (HD), and HP. In comparison to the first two therapeutic methods, HP is the most effective way [33]. However, the clearance rate of PQ in PQ-poisoned patients who received HP treatment is not reported. According to our results, the mean clearance rate of PQ treated with HP was 73 ± 15%.

PQ is absorbed quickly, but not completely, after ingestion. Animal experiments indicate that over a 1–6 hour period, PQ was absorbed poorly by the stomach and small intestine (<5%) and absorbed mostly by the jejunum [8, 34]. Moreover, PQ can distribute in high concentrations into all organs in the body, especially the lungs, heart, and kidneys [34]. PQ is also accumulated in fat and muscle which serve as important PQ reservoirs [2, 34]. Therefore, when plasma PQ concentration decreased quickly, PQ stored in tissues was released to blood. For this reason, PQ concentrations increased after first HP treatment.

The retrospective study showed early HP (<4 or <5 h after ingestion of PQ) is associated with decreased mortality in PQ-poisoned patients [13]. Our investigation revealed the survival of patients was correlated with initial PQ-concentration and early HP treatment. The patients The patients whose initial PQ-concentration was lower than 6 *μ*g/mL when decreased to less than 0.05 *μ*g/mL after received first HP treatments within 6 h were survived.

### 4.3. Prediction Model of PQ

The BP-ANN model is different from multiple logistic regression (LR) model which normally assumes the response variable should be linear in the coefficients of the predictor variables, while BP-ANN model can employ nonlinear mathematical model to process the data [35]. In this study, PQ concentrations varied in every patient and increased after HP treatment. The PQ concentration before and after HP treatment is not linear; therefore, BP-ANN model is a suitable tool for prediction.

The BP-ANN model comprised of input layer, output layer, and hidden layer. The input layer can be formed by a single feature or more various feature for a specified problem. The hidden layer receives and processes the data from the input layer, then delivers to the output layer. In this study, the PQ-concentrations of 41 patients before HP treatment were employed as variable of input layer, and the model achieved high accuracy by selecting the PQ-concentrations after HP treatment as test. When we divided PQ-poisoned patients as training group (21 patients) and test group (20 patients), the MSE was 5.76 × 10^−2^.

Consequently, we can predict the PQ concentration after HP treatment by artificial intelligence model. And if more relevant variables were selected and employed into input layer, more high accuracy would achieve. This will be very useful in emergency clinical treatment to calculate the frequency of HP treatment and what kind of therapy can be conducted.

## 5. Conclusions

HP is an effective method to remove PQ from plasma. HP results in a mean clearance rate of PQ in plasma of 73 ± 15%. A BP-ANN clearance model of PQ for HP treatment was developed and proven to be highly accurate in predicting plasma PQ concentrations after HP treatment.

## Figures and Tables

**Figure 1:** Correlation of PQ concentrations in PQ-poisoned patients before and after HP treatment.

**Figure 2:** Plasma PQ concentrations in 9 patients receiving two HP treatments within 24 hours.

**Figure 3:** The performance function of BP-ANN clearance model of PQ after reaching the training goal at epoch 157.

**Figure 4:** The measured (“+”) and predicted (“o”) plasma PQ concentrations in 41 PQ-poisoned patients after first HP treatment.

**Table 1:** Precision and accuracy of method for the determination of PQ in human plasma (*n* = 5).

Concentration (*µ*g/mL)	Measured (ng/mL)		Accuracy (%)		RE (%)	
	Intraday	Interday	Intraday	Interday	Intraday	Interday
0.08	82.80 ± 5.75	82.60 ± 7.91	6.94	9.58	3.50	3.25
0.8	816.19 ± 49.13	791.36 ± 26.51	6.02	3.35	2.02	−1.08
8	7922.45 ± 534.43	7905.97 ± 553.09	6.75	7.00	−0.97	−1.18
